The article "Surgical Design Optimization of Proximal Junctional Kyphosis" was published in 2020. Journal: J Healthc Eng.

# Surgical Design Optimization of Proximal Junctional Kyphosis

**DOI:** 10.1155/2020/8886599

**Published:** 2020-09-16

**Authors:** Li Peng, Guangming Zhang, Heng Zuo, Lan Lan, Xiaobo Zhou

**Affiliations:** ^1^West China Biomedical Big Data Center, West China Hospital/West China School of Medicine, Sichuan University, Chengdu 610041, China; ^2^School of Mathematics, Sichuan Normal University, Chengdu 610066, China; ^3^Center for Computational Systems Medicine, School of Biomedical Informatics, University of Texas Health Science Center at Houston, Houston 77030, USA

## Abstract

**Purpose:**

The objective of this study was to construct a procedural planning tool to optimize the proximal junction angle (PJA) to prevent postoperative proximal junctional kyphosis (PJK) for each scoliosis patient.

**Methods:**

Twelve patients (9 patients without PJK and 3 patients with PJK) who have been followed up for at least 2 years after surgery were included. After calculating the loading force on the cephalad intervertebral disc of upper instrumented vertebra of each patient, the finite-element method (FEM) was performed to calculate the stress of each element. The stress information was summarized into the difference value before and after operation in different regions of interest. A two-layer fully connected neural network method was applied to model the relationship between the stress information and the risk of PJK. Leave-one-out cross-validation and sensitivity analysis were implemented to assess the accuracy and stability of the trained model. The optimal PJA was predicted based on the learned model by optimization algorithm.

**Results:**

The mean prediction accuracy was 83.3% for all these cases, and the area under the curve (AUC) of prediction was 0.889. And the output variance of this model was less than 5% when the important factor values were perturbed in a range of 5%.

**Conclusion:**

Our approach integrated biomechanics and machine learning to support the surgical decision. For a new individual, the risk of PJK and optimal PJA can be simultaneously predicted based on the learned model.

## 1. Introduction

For adolescent idiopathic scoliosis (AIS) patients, orthopedic operations are employed to reconstruct the coronal and sagittal alignment to maintain the stability of spine [1]. Long posterior instrumentation and fusion surgery is often a powerful surgical treatment for spinal deformity [2, 3]. During the treatment, vertebrae are fused using pedicle screws or other combinations of devices. Such fusion treatment is intended to reconstruct spinal geometry by strong correction and derotation of the spine [4]. However, the lack of mobility in fusion segments has raised a postulation that such fusion may increase the stress in proximally cephalad spinal segments and eventually accelerate deterioration of the neighboring discs [5].

The article "Surgical Design Optimization of Proximal Junctional Kyphosis" was published in 2020. Journal: J Healthc Eng.

Powerful correction maneuvers of predominantly all-pedicle instrumentation could also result in a series of issues such as the increase of the proximal junction angle (PJA, the sagittal Cobb angle between the inferior endplate of the upper instrumented vertebra (UIV) and the superior endplate of two cephalad vertebrae ) [6]. Proximal junctional kyphosis (PJK), an abnormal kyphotic deformity involving spinal segments proximally adjacent to the fusion segments, has drawn the attention of many spine surgeons [7–9]. This frequent complication might cause regional pain, diminish quality of life, and ultimately lead to revision surgery in some severe cases [10, 11]. The generally accepted definition of PJK is described by Glattes et al. [8] that PJA is more than 10° and at least 10° greater than the preoperative measurement. The incidence rate of PJK ranges extensively from 6.0% to 45.1% [6, 8, 10, 12–14]. A retrospective review of 836 adult cases reported a higher percentage of unplanned readmission due to PJK within 90 days from surgery (51.9%) compared with other surgical complications [15].

The recent advances in computer-aided design (CAD) have been rapidly changing the landscape in scoliosis treatment procedures, improving the clinical outcomes of patients significantly as valuable models are practiced [5, 16]. Many studies biomechanically assess and evaluate the independent effects of different instrumentation variables by the finite-element method (FEM) [15, 17–21]. The difficulty mainly comes from a finite range of optimizations by manual selection. Our study focuses on designing a reliable automatic system to assist surgeons designing and preoperatively help decrease the readmission rate of scoliosis patients.

The larger difference value of preoperative and postoperative PJA (more than 5°) has been determined as a risk factor of PJK [8]. However, the individual and coupling biomechanical effects of PJA are not yet fully understood. The purpose of this paper is to predict which AIS patients have higher risks of PJK due to biomechanical factors and calculate the optimal PJA for each AIS patient. In this work, we hypothesize that inappropriate intraoperative PJA change compared with preoperation may lead to inhomogeneous distribution of loading and ultimately result in various degrees of degeneration in the cephalad intervertebral disc of UIV, and a suitable angle is beneficial for an individual patient to have a better prognosis after corrective surgery. The biomechanical information of intervertebral discs in the proximal junctional segment following spinal deformity surgery can be accurately simulated by integrating a finite-element method (FEM) with a statistical learning model.

The article "Surgical Design Optimization of Proximal Junctional Kyphosis" was published in 2020. Journal: J Healthc Eng.

## 2. Materials and Methods

This study presented an integrated approach to accurately simulate cephalad intervertebral disc behavior of the UIV for pre- and postoperation, respectively, for the purpose of optimizing the PJA for AIS patient.  Figure 1 describes the flowchart of the whole process.

This retrospective study was completed with AIS patients who undergone scoliosis correction surgery from 2013 to 2018 at West China Hospital and have been followed-up for at least 2 years to assess whether or not developing PJK. Patients were excluded if imaging information including preoperative, immediate postoperative (3–7 days after surgery) X-ray, and preoperative CT could not be obtained. Twelve cases were recruited for this biomechanical study. For each patient, the collected data involved the upper instrumented vertebral documentation, actual PJA, gender, age, and preoperative spinal computed tomography (CT). Based on the postoperative 2-year PJA, which is more than 10° and at least 10° greater than the preoperative measurement, those patients were categorized into 2 groups: PJK group and non-PJK group. In this study, we used the aforementioned study information for each patient as ground truth to confirm the patient selection.

### 2.1. Feature Extraction

#### 2.1.1. Intervertebral Disc Segmentation and Quantification

Twelve subject-specific geometries of patients were acquired using preoperative CT scans. All images were acquired with 1 mm slice intervals and a 512 × 512 acquisition matrix, and then imported into Mimics 20.0 Imaging Software (Materialise, Leuven, Belgium) for segmenting as shown in Figure 2. Initial segmentation was performed by thresholding image from 50 to 150 Hounsfield units chosen to most accurately preserve intervertebral disc geometry. Manual segmentation was employed to delineate regions, which were visible but could not be captured by automated methods. To limit the area-of-interest and reduce computational complexity, we restricted the zone to the cephalad intervertebral disc of UIV because no tissue deformations appeared in adjacent vertebrae (as shown in Figure 2(b)).

For spine corrective operation, a preprocedural plan is meaningful only if it can be accurately transferred to a patient at the time of intervention. For this reason, we applied a validated software (Surgimap, version 2.2.15.5), which could measure the degree of the curvature quickly on pre- and postprocedural standing radiographs, thus determining the influence of gravity at each vertebral level of patients with scoliosis in the upright position [22]. The severity of scoliosis can be evaluated by measuring the Cobb angle. With using strong correction of all-pedicle instrumentation, the PJA changes with reconstructing the coronal and sagittal alignment [6]. After selecting the most suitable UIV according to the scoliosis type, assuming different stress distribution of the UIV surface would derive from angular variations of PJA, and inappropriate intraoperative PJA change compared with preoperation could lead to inhomogeneous stress distribution of the upper body weight on the UIV surface and the degeneration of adjacent intervertebral disc. Usually, a virtual proximal segment correction will decrease the PJA as possible. However, due to the biomechanical properties of tissues, patients may still be at risk for PJK two years after spinal surgery because of the nonspecific PJA. Therefore, our approach addresses the need to develop a reliable process for simulating tissue behavior changes of intervertebral disc between pre- and postprocedure.

The article "Surgical Design Optimization of Proximal Junctional Kyphosis" was published in 2020. Journal: J Healthc Eng.

#### 2.1.2. Loading Force Calculation with the PJA

To study the mechanical behavior of the proximal intervertebral disc, we calculated the loading force on the tissue before and after the surgical correction. We denote *α* as the PJA at pre- or postoperation. The loading force **F** (i.e., contact force) is perpendicular to the upper surface of the intervertebral disc tissue, which is roughly equivalent to the decomposing force of the patient's gravity at this point. The decomposition angle of gravity can be estimated as *α*. Hence, **F** can be calculated by **G***∗ ***cos***α*, where **G** denotes the gravity of the body weight above UIV (as shown in Figure 2(b)) [14].

The 3D segmented intervertebral discs were first discretized into small mesh by HyperMesh (Altair, USA). To obtain high precision mesh models, they were composed of tetrahedral elements, and each element contained 4 mesh nodes tetrahedral. The mesh nodes could be classified into the boundary and free nodes; meanwhile, the boundary nodes were located in the inferior surface, which would be fixed in all degrees of freedom. We restricted the zone to the adjacent intervertebral disc of the UIV for focusing on the deformable area of interests with regard to PJK.

#### 2.1.3. Assignment of the Intervertebral Disc Properties

Intervertebral disc (IVD) tissue is composed of a nucleus pulposus (translucent gel) and an anulus fibrosus (lamellar structure), with negligible vascularization in the anulus and nucleus regions [23, 24]. Nonoriented collagen fibrils enmesh in the proteoglycan-water pulposus and are surrounded by the anulus fibrosus, a series of concentric encircling lamellae with two well-defined axes of orientation [23, 25–27]. To simplify the analysis process, we defined the intervertebral disc tissue as a linear elastic tissue with the homogenous and isotropic properties [5]. Different material parameters in terms of Young's modulus and Poisson's ratio for these two components were given by the previous work depending on biomechanical analysis and the material model as shown in Table 1 [5, 28]. These parameters were used to simulate tissue biomechanical behavior based on Hooke's law. And the heterogeneous properties of the intervertebral disc tissue will be examined in the proposed studies.

The article "Surgical Design Optimization of Proximal Junctional Kyphosis" was published in 2020. Journal: J Healthc Eng.

### 2.2. Stress Formulation

We extracted stresses as one of the biomechanical characteristics from FEM. The stress for each mesh node varies according to different components of the intervertebral disc. To obtain a distribution of stress features, we first simulated the intervertebral disc behavior responding to loading force. Denote stress features as *σ*_**i**_=*σ*(**G**_**i**_, *α*_**i**_, **E**, **v**), where *G*_*i*_ denotes the force of gravity from the body weight above UIV of the *i*th patient, and *α*_*i*_ is the pre- or postoperative PJA. Next, the stress value *σ*_*i*_ is employed as the biomechanical feature of the *i*th patient. Finally, *σ*(·) represents the stress modeled by Hooke. Here, FEM was implemented in the commercial software Altair OptiStruct. To validate our model, we loaded the pressure difference of pre- and postoperative force of one patient on his FEM model and compared the simulation results with the true geometric model of the intervertebral disc generated from postoperative CT; the absolute error of volume was 500 mm^3^, while the relative error was 2.5%, and the absolute error of average disc height on the central sagittal plane was 0.3 mm, while the relative error was 5.0%, indicating that our simplified model could save labor and machine time based on not influencing the authenticity of the FEM model [17].

To elaborate the stress variations of corresponding regions caused by the selection of PJA, stress information was evaluated on eight anatomical regions of anulus fibrous and nucleus: left anterior, left posterior, right anterior, and right posterior. The difference value Δ*σ* of before and after operation subregions max or average stress information was considered as the input biomechanical features.

### 2.3. Model Building

Surgical outcomes, i.e., PJK are closely related to the biomechanical properties such as stress induced by curvature rectification of scoliosis [11]. A two-layer fully connected network was employed to efficiently model nonlinear functions with less parameters [18, 19]. The clinical outcome *y*_*i*_/whether PJK occurred or not of *i*th patient can be modeled as the following equation:

(1) $$\begin{array}{c} y{}_{i}=g\left[\Delta \sigma {\left(G_{i},\;\alpha_{i},\;E,\;v\right)}^{1},\Delta \sigma {\left(G_{i},\;\alpha_{i},\;E,\;v\right)}^{2},\ldots ,\Delta \sigma {\left(G_{i},\;\alpha_{i},\;E,\;v\right)}^{8},\;{\text{age}}_{i},\;{\text{gender}}_{i},\;W\right], \end{array}$$

where *N* is the total number of subregions, *g*(·) is the fully connected network, and Δ*σ* denotes the max or average difference value of stress in corresponding subregions, including 16 variables. *W* is the parameter (the coefficients of the variables in *g*(·)) to be determined by minimizing an objective function as

(2) $$\begin{array}{c} \hat{W}=\underset{W}{\text{argmin}}{\left\|y{}_{i}-g\left[\Delta \sigma {\left(G_{i},\;\alpha_{i},\;E,\;v\right)}^{1},\Delta \sigma {\left(G_{i},\;\alpha_{i},\;E,\;v\right)}^{2},\ldots ,\Delta \sigma {\left(G_{i},\;\alpha_{i},\;E,\;v\right)}^{8},\;{\text{age}}_{i},\;{\text{gender}}_{i},\;W\right]\right\|}_{\text{L}2\text{ norm}}. \end{array}$$

The optimization is achieved by using Adam algorithm with calculating the exponentially weighted moving average of the gradient and then squaring the calculated gradient [20]. This optimal $\hat{W}$ is fixed for PJA simulation for new patients. The risk of PJK can be predicted from this trained model. Then, we will apply a dynamic optimization method for considering other basic clinical factors once new patients are added to the prediction model.

The article "Surgical Design Optimization of Proximal Junctional Kyphosis" was published in 2020. Journal: J Healthc Eng.

### 2.4. Clinical Outcome Prediction and the Optimal Postoperative PJA

The trained model becomes $\;y{}_{i}=g\left[\Delta \sigma {\left(G_{i},\;\alpha_{i},\;E,\;v\right)}^{1},\;\Delta \sigma {\left(G_{i},\;\alpha_{i},\;E,\;v\right)}^{2},\ldots ,\;\Delta \sigma {\left(G_{i},\;\alpha_{i},\;E,\;v\right)}^{8},\;{\text{age}}_{i},\;{\text{gender}}_{i},\;\hat{W}\right]$. When a new patient comes to the hospital, expected Y should be set to be 0, which indicates that patients will be without PJK postoperatively. $\hat{W}$ is known (from training step), and *E*,  *v* are the subregions of the intervertebral disc tissue that can be obtained from CT data by FEM from all patients. Age at surgery and gender can be collected from their demographic data. Then, we employ Adam algorithm to preoperatively estimate the idealized optimal value of $\hat{\alpha }$ for a new individual expecting no PJK as following:

(3) $$\begin{array}{c} \hat{\alpha }=\underset{\alpha }{\text{argmin}}{\left\|0-g\left[\Delta \sigma {\left(G_{i},\;\alpha_{i},\;E,\;v\right)}^{1},\;\Delta \sigma {\left(G_{i},\;\alpha_{i},\;E,\;v\right)}^{2},\ldots ,\;\Delta \sigma {\left(G_{i},\;\alpha_{i},\;E,\;v\right)}^{8},\;{\text{age}}_{i},\;{\text{gender}}_{i},\;\hat{W}\right]\right\|}_{\text{L}2\text{ norm}}. \end{array}$$

Thus, the optimal loading force $\hat{\alpha }$ can be estimated preoperatively to ensure a more successful operation.

The article "Surgical Design Optimization of Proximal Junctional Kyphosis" was published in 2020. Journal: J Healthc Eng.

To identify the most relevant features with a high degree of discrimination between PJK and non-PJK groups, we used the DX score feature selection method, whose effectiveness and efficiency have been confirmed [21]. We selected the top 5 features to perform sensitivity analysis to explore the model output variation upon a range of 5% perturbation of those important variables.

## 3. Results

### 3.1. General Information

A summary of the collected case data and the preoperative and postoperative geometric indices is provided in Table 2. Twelve cases were recruited, among which 8 were females and 4 were males with an average operation age of 16 years, ranging from 13 to 20 years and an average weight of 49 kg, ranging from 32.5 to 71 kg. The preoperative PJA in PJK and non-PJK group was 8.4° ± 2.9° (between 5.2° and 9.4°) and 6.7° ± 5.3° (between 0.9° and 18°), respectively, whereas the immediate postoperative (3–7 days after surgery) PJA was 13.0° ± 4.0° (between 9.3° and 17.2°) and 8.0° ± 4.7° (between 1.7° and 16.6°), respectively.

### 3.2. Model Performance

To complete the decision-making procedure prior to the surgery and reduce the medical cost, we proposed our reliable system for AIS patients. And to avoid overfitting, leave-one-out cross-validation was implemented to assess the accuracy of our approach. More specifically, one of all 12 patients was used for model testing while the rest for training, and these procedures were repeated until each patient had been used once as a testing sample. We evaluated the performance based on the difference between the predicted clinical results (PJK) and ground truth derived from 2 years of the follow-up study. The average prediction accuracy was 83.3% for all cases (2 out of 12). Incorrect predictions from the biomechanical and machine learning approach model for the patients are shown in Figure 3. The receiver operating characteristic (ROC) curve is illustrated in Figure 4, and the area under the curve (AUC) of prediction was 0.889.

The top 5 features with 74.3% impact percentage of all features that affected the outcome were age, max-stress variations in right anterior anulus fibrous and nucleus, and average stress variations in right anterior and left posterior nucleus. Sensitivity analysis showed that our model was stable in the sense that the output variance was less than 5% when the important factor values were perturbed in a range of 5%. The top five factors ranked by the DX score were sensitive for all patients (2.10%–4.66% upon 5% parameter perturbation) in Figure 5.

The article "Surgical Design Optimization of Proximal Junctional Kyphosis" was published in 2020. Journal: J Healthc Eng.

## 4. Discussion

This study is the first to integrate computational biomechanics and machine learning to generate clinically relevant results for surgical scoliosis treatment. A procedural planning tool was constructed to focus on predicting the risk of PJK in scoliosis patients undergoing spine surgery through computation of stress within the intervertebral disc and optimization of the PJA to prevent PJK. In clinical practice, when making a surgical plan for the new patient, we can accurately simulate his or her postoperative biomechanical behavior on proximal intervertebral disc and predict the risk of PJK and obtain the best optimal PJA with a learned model. Therefore, the decision-making procedure could be performed prior to the surgery, reducing the risk of revision related to postoperative complications.

Cases 1–9 underwent spinal corrective operation without PJK, and Cases 10–12 who had PJK after spinal corrective operation required being followed-up closely and received revision in time. Table 2 represents the predicted performance of our approach. The average of prediction accuracy was 83.3% for all cases (10 out of 12). Certain cases failed for reasons which could not be attributed to the model. For example, Case 7 failed because this patient received growing rod technique in our hospital before being treated by long posterior instrumentation and fusion surgery, which was not our research object in this model. The Case 8 might be due to vertebroplasty, a technique injecting bone cement into vertebral bodies to restore the stiffness and increasing the risk of fractures in adjacent nonaugmented vertebrae [29]. Further investigation is required to determine the biomechanical effect of vertebroplasty in developing PJK, and it is beyond the scope of this study. Our model indicated that some regions with high difference of stress before operation and after operation were observed in the PJK group. These excessive stress concentrations demonstrated that inappropriate intraoperative change of PJA would lead to a nonsynchronous variation of stress in the corresponding areas of the intervertebral disc. And the structural changes of intervertebral discs might be attributed to the inhomogeneous distribution of stress on the surface, which eventually led to an increase in the PJA. Moreover, increased PJA was associated with the clinical outcome in elderly populations [30].

Spinal instrumentation offers benefits to AIS patients whose cardiopulmonary function and growth are seriously affected by the spinal deformity [31, 32]. However, complicated issues that adversely affect surgery outcomes remain, and proper operation design may help address current challenges. For spinal instrumentation surgery, to guarantee the corrected spine is aligned together in three dimensions at the macro level; it means that there will be an inevitable risk of neglecting the detail treatment of the proximal junction region, especially PJA. For these reasons, Lee et al. [9] were the first to suggest fixing UIV + 1 if it was more than 5° to reduce the incidence of PJK after operation. However, no previous study assesses a specific and applicable PJA for each individual case with scoliosis, and our study devotes to resolve this problem. It is worthwhile to mention that simplifications and approximations have been made in the intervertebral disc FEM model construction. A more precise spine geometry may be complex and certainly time-dependent such as vertebrae and tissue degeneration, which may go beyond the biomechanical domain considered in this study. However, given that the PJK evolves primarily in the early postoperative period, the primary effects of the PJA can be estimated as mechanical modifications of the intervertebral disc such as load-stress or load-stress behaviors that in turn give rise to changes of the disk anatomical structure as function of time [16]. No tissue deformations appeared in adjacent vertebrae, and the FEM model developed in this study allowed the primary effects of the PJA to be simulated and assessed, restricting the area-of-interest to the intervertebral disc that could be considered as appropriate for this study. Belytschko et al. also indicated that material properties of the anulus obtained by direct measurement underestimated the material stiffness, and based on the disc geometry, reasonable predictions of variations of disc stiffness with vertebral level could be made [25]. Thus, the influence of material parameters associated with disc levels in surgical optimization should be the future research direction. Another simplification was that pre- and postprocedural simulations were performed on the same intravertebral disc model, which could be considered as having a limited impact on the results, because the analyses focused on the relative differences instead of the absolute numerical values of the variables.

The article "Surgical Design Optimization of Proximal Junctional Kyphosis" was published in 2020. Journal: J Healthc Eng.

The stability and accuracy of our established machine learning model have been tested and verified by the cross-validation and comprehensive sensitivity analyses. The practically applied PJA in operation and the estimation results from our model are simultaneously shown in Table 2. The optimal PJA estimation results from our model showed much consistence with the actual sizes in the non-PJK group. In addition, certain optimization results (e.g., Case 5, 6, and 8) also showed that it was unreasonable to minimize PJA blindly, and the best angle should be chosen by comprehensively considering the influence of biomechanical and demographic data. In the PJK group, the estimation results could reduce the excessive stress of the proximal intervertebral disc tissue, which might delay the early deterioration and dysfunction of proximal junctional region and lead to a favorable outcome. The estimation of Case 12 was little different compared with practically adopted PJA, and it might be caused by other nonbiomechanical problems, which were not collected and were potentially better predictors for that patient.

On account of the complexity and variability of the proximal junctional anatomy, the incidence and severity of postprocedural PJK are difficult to predict, indicating the need of a model that aid the orthopedic surgeon to select the optimal PJA that best fits the individual patient. Accurate simulation of a spinal surgery procedure based upon the integration of age and gender, the patient-specific anatomy, the biomechanical properties of the intervertebral disc tissue may serve this goal. The combination of biomechanical properties and the machine learning method substantially improved prediction of clinical results. A nonlinear FEM approach will be used to improve the accuracy in the future.

Some limitations need to be considered in this study. First, we developed finite-element models with simple linear elastic material properties for AIS patients. The anisotropy properties of the intervertebral disc tissue will be examined in the proposed studies. Second, there were very small number of patients and lacking of factors other than biomechanical and basic data. However, the current study is the first step to focus on integrating computational biomechanics and machine learning to optimize the PJA for scoliosis patients, and we will keep following up more cases in next stage.

## 5. Conclusions

In this work, we developed a procedural planning tool to predict the risk of PJK and the optimal PJA. 3D FEM models of the cephalad intervertebral disc of UIV were constructed for all patients to extract biomechanical stress information. The two-layer fully connected network was used to model the relationships between the stress information and the risk of PJK. We have integrated biomechanics and machine learning to propose a systematic approach, which devotes to support surgical decision-making by reducing the medical cost of revision after long posterior instrumentation and fusion surgery in the future.

The article "Surgical Design Optimization of Proximal Junctional Kyphosis" was published in 2020. Journal: J Healthc Eng.

## Figures and Tables

**Figure 1:** The flowchart of optimizing the surgical design of PJK. In the training phase, the machine learning model is generated. During the testing phase, the model can be used for PJA optimization based on a new patient's information.

**Figure 2:** Illustration of the biomechanical analysis process. (a) Blue rectangle means the upper instrumented vertebra (UIV), the red one is UIV + 1, and the green one is UIV + 2. (b) In the mesh data of segmented cephalad intervertebral disc of UIV, light red indicates nucleus, and dark red demonstrates anulus fibrosus; white solid lines in an enlarger X-ray represent the inferior endplate of UIV and the superior endplate of two cephalad vertebrae, respectively, and the angle formed by the intersection of them is the proximal junctional angle (PJA, *α*). (c) Loading force calculated in the previous stage on the segmented vertebra by Altair OptiStruct. (d) F, anulus fibrosus; N, nucleus; A, anterior; P, posterior; R, right; L, left.

**Figure 3:** Incorrect predictions from the biomechanical and machine learning approach model for the patients in a dataset (a and d, meshed model of the intervertebral disc; b and e, preoperative stress distribution; c and f, postoperative stress). (a–c) Case 7 was predicted to be high risk (model output, 55.6%). However, PJK was not observed until a 2-year postoperative follow-up. (d–f) The model output was 40.1% for the Case 11, in which PJK occurred 451 days after operation.

**Figure 4:** ROC curves of the two-layer fully connected network model.

**Figure 5:** Sensitivity analysis for the top 5 features ranked by DX score: age, max-stress variations in right anterior anulus fibrous (Max FAR) and nucleus (Max NAR), and average stress variations in right anterior (Avg NAR) and left posterior nucleus (Avg NPL).

**Table 1:** Material parameters of the intervertebral disc tissue [5, 28].

	Young's modulus (MPa)	Poisson's ratio
Nucleus	1.0	0.49
Anulus fibrosus	3.4	0.45

**Table 2:** Optimization performance on PJK and non-PJK group.

No.	PJK after surgery	Weight (kg)	Age at operation (year)	Gender (male: M, female: F)	Predicted results (0 = without PJK and 1 = with PJK)	Pre-PJA (°)	Applied post-PJA (°)	Optimal post-PJA (°)
1	No	56	15	M	0.425	12.4	12.9	12.6
2	No	42	17	F	0.296	5.8	7.7	6.3
3	No	64	13	F	0.345	6.9	7.8	7.4
4	No	52	20	M	0.174	5.2	9.6	3.9
5	No	37	13	F	0.270	2.4	1.7	3.4
6	No	45	16	M	0.331	18.0	16.6	18.2
7	No	71	20	F	0.556 (yes)	0.9	4.8	1.2
8	No	41	13	F	0.306	4.6	3.2	6.0
9	No	40	13	F	0.361	5.1	7.6	6.1
10	Yes	32.5	16	M	0.508	10.7	17.2	11.5
11	Yes	60	18	F	0.401 (no)	4.1	12.4	5.5
12	Yes	47.5	18	F	0.586	9.4	9.3	9.5

The article "Surgical Design Optimization of Proximal Junctional Kyphosis" was published in 2020. Journal: J Healthc Eng.

## Data Availability

The raw data used to support this study are not available and belong to West China Hospital of Sichuan University.
